# Consumption Pattern and Mental Health of Employees Based on Big Data Analysis

**DOI:** 10.1155/2022/6894141

**Published:** 2022-06-28

**Authors:** Teng Su

**Affiliations:** School of Management and Economics, Beijing Institute of Technology, Beijing 100081, China

## Abstract

With the development of big data concept and technology, big data has an important impact on human development. This paper studies the relationship between the consumption pattern and mental health of enterprise employees under the normalization of epidemic prevention and control. Starting from the consumption structure and behavior of enterprise employees, it defines the meaning of enterprise employees' consumption and the connotation of enterprise employees' health psychology and analyzes the relationship between consumption behavior and consumption psychology and the elements of enterprise employees' health psychology. Based on the change of employees' income structure and consumption patterns, this paper speculates the relationship between employees' consumption patterns and mental health, analyzes the correlation between employees' consumption patterns and mental health through a questionnaire survey, and calculates the Correlation Clustering statistical results. It plays an important role in building a good enterprise staff consumption culture under the normalization of epidemic prevention and control and effectively realizes the significance of purifying the social consumption environment.

## 1. Introduction

During the epidemic period, not only the economic situation changed but also the behavior and attitude of global consumers had changed dramatically. The purpose of studying consumer psychology also includes meeting the psychological and physiological requirements of consumers, developing appropriate strategies for consumer services, and providing strong support for the protection of consumer interests. In daily life, in addition to learning, work, and entertainment, satisfying the desire of consumption leads to pleasure and happiness. The study of consumers' psychology and behavior mode can better meet the consumption pleasure of consumers. In consumer psychology, the study of consumers' subjective feelings, experience, and satisfaction is a necessary prerequisite for formulating service strategies. How to protect the employees at the grassroots level, what changes have taken place in people's consumption mentality, and what is the difference between the consumer market and the past? These problems have become the focus of people's attention. Therefore, from the perspective of normalization of epidemic prevention and control, this paper studies the correlation probability between employees' consumption patterns and mental health. In general, risk can be expressed as a function of the probability of events and their consequences [1–3], namely,

(1) $$\begin{array}{c} R=F\left(P,C\right), \end{array}$$

where *R* is the epidemic risk degree; *P* is the probability of changes in consumption patterns of enterprise employees after the epidemic; and *C* is the consequences of changes in consumption patterns and mental health of corporate employees after the epidemic.

The occurrence probability of this kind of bad event is described by the epidemic risk degree in the above function, so the risk is always associated with the loss. Therefore, the loss is regarded as the starting point of the research on the correlation between the consumption style and mental health of enterprise employees, that is, the concept of dosage is used to specify the risk [4, 5]. The probability of loss refers to the probability or opportunity of loss in a certain period of time. In a more popular sense, risk actually represents an uncertainty that is always associated with potential losses.

Mental health problems are the result of the comprehensive action of various factors. There are many reasons for the increase of employees' psychological problems, mainly including social environmental factors, enterprise environmental factors, family environmental factors, and employees' psychological factors. Employees' mental health problems will inevitably be reflected in daily work, study, life, social interaction, etc., and will have a negative impact on work efficiency, work stability, and even the harmonious development of the whole society. Enterprise managers and even the whole society should incorporate the adjustment and release of employees' psychological problems into their daily management work and strive to improve the mental health level of employees. The main countermeasures to solve the mental health problems of employees are paying close attention to their mental health, improving their social adaptability, striving to create a good environment conducive to the mental health of employees, and reducing stressors.

Therefore, in the research on the relationship between employees' consumption patterns and mental health, we can follow the idea of empirical research on definition behavior and psychological analysis. Then, the definition of a healthy personality of employees is given, and the constitution of the healthy personality is analyzed. Finally, using the change of employees' income structure and employees' consumption patterns, we speculate the relationship between employees' consumption patterns and mental health and calculate the Correlation Clustering statistical results. The flow chart of this paper is shown in Figure 1.

## 2. Materials and Methods

### 2.1. Consumer Definition

Consumption is a kind of economic relationship. In the case of consumption activities, employees' consumption includes work and production needs, transportation needs, living environment needs, and material needs. An earlier meaning of consumption is a process of spending money to meet one's own needs [6–9]. And, consumer behavior is a kind of external activity driven by consumer psychology, which may be practical or spiritual things and may include now paid music, paid TV programs, food, daily necessities, and so on.

In the process of social development, the study of consumer behavior is not limited to the field of psychology, but closer to the field of sociology.

This paper discusses the consumption pattern of enterprise employees under the normalization of epidemic prevention and control, discusses consumption level and consumption structure of enterprise employees before and after the epidemic, and analyzes the influence of enterprise employees' healthy psychological environment on consumption behavior, so as to make a comprehensive analysis of enterprise employees' daily life and social economy.

### 2.2. Analysis of Consumption Behavior and Consumption Psychology of Enterprise Employees

The consumption psychology of enterprise employees is a kind of inner emotional process of spending money and time to obtain various goods. What we call the desire to buy certain things and the psychological comfort after purchasing certain things all belong to the consumption psychology of enterprise employees [10–15]. At present, employees in enterprises generally have the following situations when they consume.

The first is task-based consumption behavior. When purchasing certain goods, it is because of the requirements of the leaders or the company, including but not limited to customizing the company's uniform clothing, raising funds for group construction, and requiring some office software or office equipment needed for work. In these cases, most employees are reluctant to consume.

Second, the consumption behavior of the company's employees is not the consumption behavior required by the company, but the consumption behavior caused by the comparison with colleagues. This includes, but is not limited to, buying clothes, accessories, lunches, and things better than what colleagues buy. In comparative psychology, most consumption is the spontaneous behavior of employees. Third, the employees of the company have a relatively pure consumption psychology, which is based on a real demand for goods. After consumption, the company's employees can get psychological comfort.

The abovementioned enterprise employees' consumption behavior is based on employees' consumption psychology, which is a predictable activity. In order to study the relationship between the consumption pattern and mental health of enterprise employees under the normalization of epidemic prevention and control, it is necessary to study the consumption psychology. The consumption behavior and consumption psychology of enterprise employees complement each other and are inseparable [16, 17].

Based on the observation and analysis of employees' consumption behavior, this paper uses the symbolic consumption theory, conspicuous consumption theory, and fashion consumption theory of consumption sociology to reveal the change trend of employees' consumption psychology.

### 2.3. Consumerism

How to evaluate the relationship between consumer behavior and mental health? Healthy consumption psychology can make the consumption behavior of enterprise employees more reasonable, and at the same time, healthy psychology can make the consumption behavior of enterprise employees more clear, can weaken the enterprise employees' desire of comparison and excessive shopping desire, also make the consumption behavior of enterprise employees more in line with China's national conditions, and advocate the consumption concept of diligence and thrift.

### 2.4. Analysis on the Construction of Healthy Personality

The mental health of the employees needs the assistance of healthy personality. Therefore, we need to clarify the connotation of the healthy personality of the employees. Healthy personality is a good character, which includes no aggressive personality, no violence, sincerity, and good treatment, which makes the employees of enterprises have a more ideal personality [18–21]. In order to analyze the mental health and consumption behavior of enterprise employees, it is necessary to analyze the definition of the healthy personality and the constitution of the healthy personality of the employees.

### 2.5. The Definition of Healthy Personality of Enterprise Employees

The healthy personality of enterprise employees is basically consistent with other personality, so it has not been clearly defined. For the convenience of this study, this paper can define the healthy personality of enterprise employees as a comprehensive ability that enterprise employees can adapt to the environment and solve problems when they encounter various challenges, difficulties, or major changes in the company or work [22–24]. Such capabilities include the following:

1. How to regulate personal emotions and not bring them into work?
2. How to improve the working environment and choose a favorable way to solve the difficulties?
3. How to mobilize the enthusiasm of individual employees when they are tired or repetitive?

This is a kind of continuous ability, or a kind of psychological adaptability. For enterprise employees, healthy personality can make employees have a strong ability to resist pressure, make them have a certain sense of security without needing others, make them release kindness to enterprise employees, make them strive to live their own life, help them do their own work well, make them observe the environment correctly and objectively, and adapt to the environment. This kind of personality can make enterprise employees less likely to panic when they encounter emergencies which leads to abnormal consumption behavior of enterprise employees.

Even people with a perfectly healthy personality can acquire mental health concerns, and it is crucial to understand how the concept of a healthy personality and the existence of mental health issues has been conceptualized. A person with a healthy personality, such as good working abilities and a high moral character, might yet suffer from mental health problems.

### 2.6. The Constitution of Healthy Personality of Enterprise Employees

This paper analyzes how to develop a healthy personality in enterprise employees on the basis of obtaining the consumption psychology and behavior of enterprise employees.

First of all, the most important thing for an enterprise is its employees' working ability. Frankly speaking, it can bring benefits to the company. Therefore, the most important thing for an enterprise employees' healthy personality is their working ability. Ability includes two aspects: one is self-ability and the other is the potential ability of enterprise employees, that is, learning to improve their own ability, which is the cornerstone of healthy personality of enterprise employees.

Secondly, the moral character of employees is also one of the important factors. In the process of work, enterprise employees need to follow their heart and be compassionate. Excellent enterprise employees should not only pay attention to current affairs, but also try their best to help others [25]. Therefore, excellent moral character plays an important role in the healthy personality of employees.

Therefore, good temperament cultivation is also an important part of the healthy personality of enterprise employees. The elements that constitute the healthy personality of enterprise employees are of multilevel, and there is an organic systematic connection between them. They have an inseparable nature in the complete personality structure. They are intertwined, interdependent, interrelated, and interactive, and together constitute the overall healthy personality of enterprise employees.

## 3. Analysis on the Relationship between Consumption Style and Mental Health of Enterprise Employees

### 3.1. Analysis on the Change of Enterprise Employees' Consumption Patterns under the Normalization of Epidemic Prevention and Control

In order to verify the relationship between consumption patterns and mental health of enterprise employees under the normalization of epidemic prevention and control, firstly the consumption patterns and sources of funds of enterprise employees are collected. This paper randomly selects 3000 employees from 10 enterprises in a city to analyze the sources of consumption funds of employees in different enterprises in 2018, and the results are shown in Table 1.

Analysis of Table 1 shows that due to the different family conditions, wages, consumption patterns, and consumption concepts of enterprise employees, the sources of consumption funds for enterprise employees are different. Among the 3000 employees, 986 used their wages for consumption, accounting for 32.87%, 523 used their credit cards for consumption, accounting for 17.43%, and 1062 used their flowers, Mayi Pay, which is a consumer credit product launched by Ant Financial, for consumption, accounting for 35.40%. The overall analysis of the above details shows that Huabei and credit card are the main ways of enterprise employees' capital consumption, which shows that with the development of network technology, people's living conditions and consumption ideas have changed.

However, the current outbreak has changed the consumption mode of enterprise employees again. Therefore, this paper makes a return visit to the 3000 employees in 2020 and analyzes the changes of consumption mode of enterprise employees under the normalization of epidemic prevention and control, and the results are shown in Table 2.

According to the analysis of Table 2, in 2020, 1868 employees of 3000 enterprises spent their wages for consumption, accounting for 62.23%, 298 employees used their credit cards for consumption, accounting for 9.93%, and 663 employees spent their money for consumption, accounting for 22.10%. 148 people spent through bank loans, accounting for 4.93%. 23 people consumed in other ways, accounting for only 0.07%. Comparing Tables 1 and 2, it can be seen that under the influence of the epidemic in 2020, the number of employees taking wages as the main source of consumption increased from 986 to 1868, accounting for 62.23% from 32.87%. At the same time, in 2020, the number of employees who used credit card and E-Payment as the main consumption mode was significantly reduced, indicating that the epidemic has affected the consumption psychology and mental health of enterprise employees.

### 3.2. The Consumption Quota of Enterprise Employees under the Normalization of Epidemic Prevention and Control

In order to further study the consumption situation of enterprise employees under the normalization of epidemic prevention and control, 3000 employees with different salaries were selected for consumption analysis and the consumption funds of employees of different enterprises in 2018 were obtained. The results are shown in Table 3.

By analyzing Table 3, we can see the consumption situation of employees in 2018. For the employees with a salary of 0–3000 yuan, one-tenth of them are paid in the range of 10000–15000 yuan and about 47% of them are paid in the range of 3000–10000 yuan. This shows that half of the employees' wages are below 10000 yuan before the outbreak of the epidemic. According to the analysis of the way of consumption of their employees, 59% of the employees who earn less than 3000 yuan are paid by WeChat, Alipay, and other electronic payment methods. 31.2% of the employees spend their money through flower and credit cards, and only 9.8% of their employees are paid by cash. Of the employees earning 8000–10000 yuan, 56% were paid by WeChat, Alipay, and other electronic payment methods. 20% of the employees were paid using Huabei and credit cards, and 24% of the employees were paid by cash. Comparing the two kinds of employees, the higher the salary, the smaller the proportion of people who use overdue consumption such as Huabei and credit card. This is also true for employees with an income of 10000–15000 yuan or more.

In order to compare the consumption situation of enterprise employees under the normalization of epidemic prevention and control, the consumption situation and income situation of 3000 enterprise employees in 2020 were collected and the consumption funds of employees were obtained as shown in Table 4.

According to the analysis of Table 4, under the influence of the epidemic, the income of these 3000 employees has changed. The number of employees whose wages were 0–3000 yuan increased from 1000 to 1200, and the number of employees whose wages were 10000–15000 yuan or more decreased by 380. This shows that the epidemic environment has affected the wages of most enterprise employees and changed their living or working environment. Compared with 2018, 81.83% of the employees who earned 0–3000 yuan were more dependent on Alipay and WeChat's electronic payment methods and the number of people who used advanced consumption methods such as Huabei and credit cards decreased from 312 to 122, which indicated that the epidemic environment affected the consumption patterns of most employees. That is to say, the epidemic prevention and control has a certain impact on the consumption style and mental health of employees.

### 3.3. Cluster Statistical Analysis of the Correlation between Consumption Patterns and Mental Health

The correlation between consumption patterns and mental health of enterprise employees under epidemic prevention and control can be obtained through cluster statistics. This paper selects the above experimental data to obtain the correlation.

In Table 5, when *p* < 0.001, it is indicated by “^*∗∗∗*^” which indicates that there is a statistically significant correlation between employees' consumption style and mental health under the epidemic prevention and control. We have three ways of employee consumption: type I (electronic payment), type II (advanced consumption), and type III (cash). In this paper, consumption skills can be described as the ability of employees to spend money and time to get what they need. Consumption skills fundamentally determine whether consumers can get satisfaction from the consumption of products and services, that is, whether the purpose of consumption can be achieved. It can be seen from Table 5 that there is a certain correlation between employees' consumption patterns and mental health under the epidemic prevention and control, and nearly half of the employees prefer electronic payment. Any kind of consumption activity includes both the psychological activity and the consumption behavior of consumers. Accurately grasping the psychological activities of consumers is the premise of accurately understanding consumer behavior. Consumption behavior is the external expression of consumer psychology, which is more realistic than consumer psychology.

In the future, based on big data mining technology, an analysis system construction strategy for consumer characteristics can be proposed. Through the effective mining and analysis of massive data, the market prospect and consumer purchase behavior of products can be predicted, so as to support auxiliary enterprises to develop reasonable marketing strategies.

## 4. Conclusion

In the research on the relationship between employees' consumption patterns and mental health, we can follow the idea of empirical research on definition behavior and psychological analysis. Then, the definition of a healthy personality of employees is given and the constitution of the healthy personality is analyzed. Finally, using the change of employees' income structure and employees' consumption patterns, we speculate the relationship between employees' consumption patterns and mental health and calculate the Correlation Clustering statistical results.

In order to study the relationship between consumption patterns and mental health of enterprise employees under the normalization of epidemic prevention and control, this paper analyzes the correlation between consumption patterns and mental health from three experiments: the income structure of enterprise employees, the correlation between income levels and consumption patterns of enterprise employees, and cluster statistics:

1. Under the influence of the epidemic, the number of enterprise employees who take wages as the main source of consumption increased by 882, accounting for 62.23%. At the same time, the number of enterprise employees using credit card and flower chant as the main consumption mode decreased significantly, indicating that the normalization of epidemic prevention and control has affected the consumption psychology and mental health of enterprise employees.
2. Compared with the preepidemic situation, 81.83% of the employees who were paid 0–3000 yuan in the enterprise were more dependent on Alipay and WeChat's electronic payment methods and the number of people using advanced consumption decreased by 190. The epidemic prevention and control had a certain impact on the way of consumption and mental health of employees.

## Figures and Tables

**Figure 1:** Flow chart of research ideas on the correlation between employees' consumption patterns and mental health.

**Table 1:** Proportion of capital sources of employees' consumption in 2018.

The source of enterprise employees' consumption funds	Number/person	Proportion/%

Wages	986	32.87%
Credit card	523	17.43%
Flowers	1062	35.40%
Bank loans	426	14.20%
Other	3	0.01%
Total	3000	100%

**Table 2:** Proportion of capital sources of enterprise employees' consumption in 2020.

The source of enterprise employees' consumption funds	Number/person	Proportion/%

Wages	1868	62.23%
Credit card	298	9.93%
Flowers	663	22.10%
Bank loans	148	4.93%
Other	23	0.07%
Total	3000	100%

**Table 3:** Consumption analysis of employees in different enterprises in 2018.

Salary range (yuan)	Consumption pattern of enterprise employees			
	Huabei, credit card	Cash	WeChat, Alipay	Total number

0–3000	312	98	590	1000
3000–5000	385	215	160	760
5000–8000	58	94	88	240
8000–10000	100	120	280	500
10000–15000	50	155	95	300
Over 15000	15	87	98	200

**Table 4:** Consumption analysis of employees in different enterprises in 2020.

Salary range (yuan)	Consumption pattern of enterprise employees			
	Huabei, credit card	Cash	WeChat, Alipay	Total number

0–3000	122	96	982	1200
3000–5000	285	220	45	550
5000–8000	45	58	127	230
8000–10000	189	301	310	800
10000–15000	4	21	95	120
Over 15000	12	33	55	100

**Table 5:** Correlation between consumption patterns and mental health after cluster analysis.

Consumption level/month	Type I	Type II	Type III	*F* value

0–500	55.823 ± 1.66	43.935 ± 1.08	55.842 ± 7.16	63.554
500–1000	53.832 ± 1.88	23.845 ± 1.31	55.643 ± 2.62	231.543^*∗∗∗*^
1000–2000	14.411 ± 2.16	53.653 ± 2.26	55.643 ± 4.51	164.553^*∗∗∗*^
3000–5000	22.563 ± 6.43	76.753 ± 4.86	55.635 ± 1.99	431.542^*∗∗∗*^
5000–8000	52.521 ± 3.11	23.532 ± 2.56	55.342 ± 1.97	643.231^*∗∗∗*^
8000–15000	54.376 ± 4.32	53.643 ± 4.16	55.654 ± 1.76	743.321^*∗∗∗*^
15000–20000	65.887 ± 3.13	35.326 ± 3.32	55.133 ± 1.54	234.664^*∗∗∗*^
20000–50000	54.896 ± 4.21	64.642 ± 5.33	55.568 ± 1.64	243.431^*∗∗∗*^
Over 50000	32.843 ± 2.16	66.532 ± 6.16	55.642 ± 1.31	532.321^*∗∗∗*^
Class size	46.25%	24.21%	29.54%	—

## Data Availability

The datasets used and/or analyzed during the current study are available from the author on reasonable request.
